This article has been retracted.

# Prognosis Evaluation of MRI Combined with Magnetic Resonance Myelography on Lumbar Disc Herniation after Transforaminal Endoscopic Discectomy

**DOI:** 10.1155/2022/2895575

**Published:** 2022-02-21

**Authors:** Yi Jiang, Rujun Zuo, Shuai Yuan, Jian Li, Chang Liu, Jiexun Zhang, Ming Ma, Dasheng Li, Yong Hai

**Affiliations:** ^1^Department of Orthopedics, Beijing Chao-Yang Hospital, Capital Medical University, Chao-Yang District, Beijing 100020, China; ^2^Department of Orthopedics (Minimally Invasive Spine Surgery Branch), Beijing Haidian Hospital (Haidian Section of Peking University Third Hospital), Hai-Dian District, Beijing, China; ^3^Department of Radiology Department, Beijing Haidian Hospital (Haidian Section of Peking University Third Hospital), Hai-Dian District, Beijing, China

## Abstract

**Objective:**

This study sets out to investigate the role of magnetic resonance imaging (MRI) combined with magnetic resonance myelography (MRM) in patients after percutaneous transforaminal endoscopic discectomy (PTED) and to evaluate its value in postoperative rehabilitation.

**Methods:**

The clinical date of 96 patients with lumbar disc herniation (LDH) after PTED was retrospectively analyzed. The enrolled patients were divided into MRI group (*n* = 32) and MRI + MRM group (*n* = 64) according to whether MRM was performed. The nerve root sleeve (morphology, deformation) and dural indentation, intervertebral space height (ISH), intervertebral space angle (ISA), degree of pain (Visual Analogue Scale (VAS)), vertebral function (Japanese Orthopaedic Association (JOA)), and long-term recurrence were compared between the two groups.

**Results:**

Compared with the MRI group, the MRI + MRM group better displayed nerve root morphology, sheath sleeve deformation, and dural indentation. Both MRI and MRI + MRM showed ISH and ISA changes well. Compared with the MRI group, the MRI + MRM group had a significantly lower VAS score for lumbar and leg pain, a significantly higher JOA score, and a significantly lower 2-year recurrence rate.

**Conclusion:**

MRM combined with MRI is more beneficial to improve the prognosis of LDH patients after PTED.

## 1. Introduction

Lumbar disc herniation (LDH), a common disease in clinic, is caused by a sedentary lifestyle and lumbar intervertebral disc degeneration with age, which predispose intervertebral disc annulus fibrosis to injury by compression, resulting in the protrusion of the nucleus pulpous into the spinal canal [1, 2]. If the protruding nucleus pulpous compresses the dural sac or nerve roots, it will cause pain in the patients' back and legs, seriously affecting their quality of life [3]. Currently, surgery is mainly used for LDH patients with poor response to conservative treatment. However, traditional discectomy plus laminotomy is more invasive and results in slower recovery [4]. With the introduction of minimally invasive concepts such as small wound and fast recovery, as well as the rapid development of medical technology, percutaneous transforaminal endoscopic discectomy (PTED) has been widely used in clinical practice and achieved encouraging therapeutic effects [5, 6]. Moreover, LDH patients have a certain risk of recurrence after surgery [7]. Therefore, it is of great significance to monitor the postoperative recovery of intervertebral discs and nerve roots and predict the recovery degree of patients, so as to guide clinical follow-up treatment [8]. At present, magnetic resonance imaging (MRI) technology has been widely used in the diagnosis of LDH, as the sagittal T 1 weighted image (T1WI), T2WI, and axial T2WI signals can clearly show the shape of the intervertebral disc, which has important clinical guiding significance for the measurement of intervertebral space height (ISH) and the judgement of postoperative residual intervertebral disc [9]. However, because of the discontinuous scanning and thick scanning layers, MRI cannot accurately show the anatomical structure around the nerve roots in the spinal canal, which makes it difficult to determine whether the nerve root is still compressed [10, 11] or abnormal in shape, affecting doctors' judgment of the degree of postoperative recovery. Therefore, looking for an imaging examination that can accurately reflect the postoperative nerve root compression and deformation is of great importance in clinical treatment of LDH.

Magnetic resonance myelography (MRM) is a noninvasive water imaging technique extensively used in clinical practice. Without the need for contrast medium and lumbar puncture, MRM can use fat suppression techniques and fast spin echo sequences to obtain high-quality images of the spinal cavity [12]. During continuous scanning, MRM can highlight the long T2 signal of cerebrospinal fluid (CSF) and improve the contrast of CSF signal, thus focusing on displaying the dural sac and nerve root sheath sleeve enclosing the CSF [13]. At the same time, the fat suppression technology can reduce the signal intensity of fat and other tissues. Finally, through coronal continuous scanning, high contrast images of the spinal cord structure can be obtained with high spatial resolution, which can clearly display images of the dural sac, spinal cord, and nerve roots [14]. On MRM images, the two sides of the nerve root sheath sleeve were mainly presented with symmetrical beak-like protrusions. Once the intervertebral disc protrudes into the spinal canal, MRM can clearly show the anatomical relationship between the disc, dural sac, and nerve root and clarify the compression of nerve root and spinal cord [15]. When the nerve root is compressed, the flow of CSF in the nerve root sheath will be reduced or even blocked, resulting in weakened or loss of T2WI signal on MRM, which contributes to a more realistic and reliable display of nerve root compression. In this study, we compared the imaging effects of MRI and MRM on the lumbar intervertebral disc and spinal cord surgical levels during postoperative rehabilitation of patients with PTED, aiming to explore their guiding role in clinical follow-up treatment.

## 2. Materials and Methods

### 2.1. Selection of Research Participants

The clinical and imaging data of patients with LDH treated in our department from January 2017 to January 2019 were retrospectively analyzed, and those who met the experimental standard were selected as the research participants. Inclusion criteria are as follows: (1) complete clinical and imaging data, including lumbar X-ray, MRI, or MRM; (2) single-level LDH at the L4/L5 or L5/S1 level; (3) those who underwent PTED; (4) age range 30–50 years old; and (5) those with good clinical compliance that could cooperate with the follow-up. Exclusion criteria are as follows: (1) history of lumbar spine surgery, (2) lumbar spinal stenosis, (3) spinal or spinal cord tumor, (4) spinal deformity, and (5) severe osteoporosis. A total of 96 patients were included in the study. Patients were divided into MRI group (*n* = 64) and MRI + MRM group (*n* = 32) according to whether lumbar MRM was performed after operation. The clinical data of patients are shown in Table 1. All the enrolled patients and their guardians gave informed consent to the study and voluntarily signed informed consent. The study has been supported and approved by the Ethics Committee of our hospital.

### 2.2. Postoperative Lumbar MRI or MRM Examination

(1) MRI examination: the 3.0T Signa HDxt scanning system (GE Company, USA) was used to routinely scan the lumbar vertebra and the sagittal position of bilateral vertebrae. T 1 weighted image (T1WI) parameters are as follows: TR 700 ms, TE 10 ms, layer thickness 4.5 mm, layer spacing 0.9 mm, and acquisition times 2; T2WI parameters are as follows: TR 3700 ms, TE 120 ms, layer thickness 4.5 mm, layer spacing 0.9 mm, and acquisition times 2. An axial scan of the L4-S1 intervertebral discs was performed with the T2WI parameters as follows: TR 4500 ms, TE 120 ms, layer thickness 5.0 mm, layer spacing 0.9 mm, and acquisition times 3 [16, 17]; (2) MRM examination: the anterior and posterior edges of the dural sac on the coronal plane were scanned using three-dimensional (3D) fast asymmetric spin-echo (FASE) sequences with the scanning parameters of TR 8000 ms, TE 120 ms, layer thickness 1 mm, and acquisition times 1. Fat suppression technology was used to reduce the systemic tissue signal and highlight the CSF signal, thus clearly outlining the spinal cord structure. Sagittal imaging was performed with layers 23-40, adjustment matrix 384 × 384, adjustment vision 300 mm × 300 mm, and scanning time 3.5-6 min. The maximum intensity projection method was used to reconstruct the source image, and the rotation axis was in the head-foot direction [18, 19]. MRI and MRM images were blindly reviewed by two experienced radiologists (Figure 1).

### 2.3. Epidural Indentation and Nerve Root Deformity at the Operative Level on MRI and MRM

The intervertebral disc protruding into the spinal canal compresses the dural sac, creating an indentation whose length and depth are positively correlated with spinal cord compression. Therefore, observing the epidural indentation is helpful in determining the degree of spinal cord compression. The sagittal diameter and longitudinal axis of the epidural indentation were measured and recorded on MRI and MRM images. Spinal nerve roots can transmit body temperature, pain, and proprioception, and if they change course or become deformed by compression, they can induce nerve conduction block, causing clinical symptoms. Therefore, observing the running course of nerve roots can help to maintain nerve compression. In this study, we mainly observed and recorded the changes in the morphology and course of nerve root sheath sleeve on MRI and MRM.

### 2.4. ISH and Intervertebral Space Angle (ISA) of Intervertebral Space at the Operative Level on MRI and MRM

Postoperative maintenance of the intervertebral disc space is of great significance to prevent lumbar disc recompression. In this study, the ISH was measured according to imaging data. The ISA reflects the curvature of the lumbar spine and the compression force on the intervertebral disc. During data measurement, the angle is positive if the parallel line of the superior and inferior border of the intervertebral space intersects in front of the lumbar spine and negative otherwise.

### 2.5. Observation of Postoperative Lumbocrural Pain and Spinal Function

The Visual Analogue Scale (VAS) was used to evaluate the waist and leg pain degree of patients before and after operation. The pain was divided into 11 levels (0-10 points), and the pain degree increases with the score [20]. The Japanese Orthopaedic Association (JOA) score was used to evaluate the lumbar functional activity of patients. The scale included 4 categories and 8 items, with a total score of 29 points. The higher the JOA score, the better the recovery of lumbar functional activity [21].

### 2.6. Patient Follow-Up

All patients were followed up every 3 months for two years by means of outpatient visits, telephone, etc., so as to observe the recurrence of LDH at the operative level. Recurrence was diagnosed with ipsilateral or contralateral disc herniation 6 months after surgery. In addition, the stability of lumbar vertebrae was observed on imaging.

### 2.7. Statistical Analysis

All data were statistically analyzed using the SPSS17.0 software, and image rendering was performed using GraphPad Prism 5.0. The enumeration data such as gender (*n*/%) were analyzed by the chi-square test. The quantitative data such as age were expressed as (^−^*χ* ± s). The comparison between groups was performed by the independent samples *t*-test, the comparison within groups before and after treatment was performed by the paired *t*-test, and the comparison among multiple groups was performed by univariate analysis. *P* < 0.05 was considered statistically significant.

## 3. Results and Discussion

### 3.1. MRI and MRI + MRM Observation of Nerve Root Sheath Sleeve

In LDH patients with nerve root compression, MRI images will show signs of nerve root sleeve deformation, deformation, or even truncation. Therefore, clear observation of postoperative nerve root compression is helpful to predict the prognosis of patients and guide further clinical treatment. In this study, we found that MRI + MRM could better detect the nerve root deformation and sheath sleeve deformation after surgery, while MRI detection was relatively easy to miss the above diagnosis (Figure 2), suggesting that the fat suppression technology of MRI + MRM could assist doctors to better observe nerve root compression.

### 3.2. Observation on the Changes of Epidural Indentation on MRI and MRI + MRM

Intraspinal disc compression of the dural sac will lead to epidural indentation on the image. The observation of compression degree can help to judge the extent of spinal cord compression. After treatment, the epidural indentation of patients was significantly reduced, suggesting that PTED could significantly relieve the compression caused by intervertebral disc herniation. Among them, the radius vector and longitudinal axis of the dural sac on MRI + MRM images were higher than those on MRI (*P* < 0.05) (Figure 3), suggesting that MRM could better display CSF by using fat suppression technology, so as to achieve the purpose of clinical myelography. Therefore, MRI + MRM could better observe the compression of the dural sac and guide doctors to better carry out treatment.

### 3.3. Measurement of ISH Loss and ISA Change on MRI and MRI + MRM

The loss of intervertebral space after PTED is easy to occur, which is related to the loss of nucleus pulpous components caused by radiofrequency thermocoagulation hemostasis and the destruction of annulus fibrosis during surgery. The observation of ISH loss degree is helpful for prospective evaluation of LDH recurrence. In this study, there was no significant difference in the detection of ISH loss between the two groups (*P* > 0.05) (Figure 4(a)). The measurement of ISA can help to determine the curvature of adjacent vertebrae and predict the recurrence of lumbar disc protrusion. In this study, no significant difference was found in ISA between MRI + MRM and MRI (*P* > 0.05) (Figure 4(b)). The above results suggested that both MRI + MRM and MRI could better display ISH loss and ISA changes.

### 3.4. Comparison of Lumbocrural Pain Degree and Lumbar Function Recovery

The degree of postoperative lumbar and leg pain can significantly reflect the outcome of surgery, as well as the recurrence of postoperative LDH and spinal nerve root compression. After surgery, the lumbocrural pain was significantly relieved in both groups with significantly decreased VAS scores (*P* < 0.05), and the long-term VAS score decrease in the MRI + MRM group was more obvious (*P* < 0.05) (Figure 5(a)), suggesting better postoperative recovery of patients in the MRI + MRM group. In terms of lumbar motion function, patients in both groups recovered significantly after surgery, and the long-term JOA score of the MRI + MRM group was higher (*P* < 0.05) (Figure 5(b)). These results suggested that MRI + MRM could better display spinal cord and nerve root compression and guide doctors to take corresponding treatment measures earlier, thus better reducing patients' pain and restoring lumbar spine mobility.

### 3.5. Comparison of Recurrent LDH and Lumbar Stability at the Operative Level

During the 2-year follow-up period, patients in the MRI group were more likely to experience LDH recurrence, and the incidence of instability at the operative level was 17.19%, which was higher than that of 6.25% in the MRI + MRM group (Figure 6(a)). The above results suggested that MRI + MRM could provide clinicians with better early warning information, allowing for early targeted treatment measures after PTED to avoid the recurrence of LDH and maintain lumbar instability (Figure 6(b)).

## 4. Discussion

LDH is a common disease in orthopedics. Due to the increase of sedentary office workers and learners in modern life, the LDH incidence rate is increasing year by year, with an emerging trend of the disease at younger ages [22]. At present, surgery is indicated in LDH patients if regular massage, traction, and other conservative treatment cannot alleviate waist and leg pain [23]. With the advances in science and technology, as well as the innovation of medical technology, there are more options for surgical treatment of LDH, such as PTED [24]. Besides, the concept of rapid rehabilitation is increasingly popularized in modern surgical treatment. PTED has the advantages of minimally invasiveness, short operation time, and fast recovery, which is in line with the concept of rapid rehabilitation [25, 26]. Therefore, PTED has been widely used in the treatment of LDH patients. At present, close follow-up observation of nerve root decompression and recovery in PTED patients are helpful for clinicians to determine the treatment plan and carry out targeted and individualized treatment [27]. Therefore, finding an examination method with small injury and high accuracy can significantly improve the doctor's understanding of the recovery of patients after PTED and help to formulate better treatment plans.

MRM, also known as magnetic resonance hydrography, can better highlight the T2 signal of spinal fluid than MRI, while more effectively suppressing the influence of fat tissue and other tissues [28]. As both the spinal cord and nerve roots are infiltrated in CSF, the running course and compression of the nerves can be observed clearly on MRM images. After PTED, the patient's normal physiological and anatomical structure is relatively disordered due to the operation, and MRI shows discontinuous scans with thick scanning layers [29]. Therefore, it is difficult to observe the complete spinal nerve root deviation on MRI, which affects doctors' judgment of postoperative nerve root decompression. On the other hand, the use of contrast agent for observation may cause certain trauma to patients, accompanied by a risk of allergy. While in virtue of advantages such as noninvasion and no need for contrast agent, MRM can solve the above problems in clinical examination. This is particularly true for patients with L 4/5 herniation; it is difficult to distinguish nerve root compression on MRI because the initial site of the L5 nerve root is thinner and there is less fat space around the nerve roots after separation from the spinal cord [30]. Besides, MRI is difficult to determine scar compression and postoperative arachnoid adhesion, while MRM has high resolution and can be reconstructed in three dimensions, which can assist clinicians to observe nerve roots from many angles [31] and help to guide postoperative rehabilitation. Some previous studies have also shown that MRM has a certain clinical application value in some orthopedic surgeries. For example, Lee et al. [15] pointed out that MRM has a high sensitivity in the preoperative diagnosis of intervertebral foramen or extraforaminal entrapment at the lumbosacral junction, and the sensitivity is comparable to that of computed tomography. Pui and Husen [32] also reported that MRM is beneficial to the observation of dural sac and root cannula and has a certain diagnostic value in spinal canal stenosis and intervertebral disc herniation.

In the examination of postoperative nerve root compression, it was found that the detection rate of MRM for nerve root deformation and sheath sleeve deformation was significantly higher than that of MRI, which suggested that MRM could better detect residual nerve root stimulation in postoperative patients and better evaluate the surgical effect. And in the observation of dural sac indentation, MRM was more sensitive to changes in the length of indentation, which could better evaluate the relief of postoperative spinal cord compression. The main reason may be that the discontinuous scan and thicker scanning layer of MRI affected the observation of lumbar nerve root movement, especially at the L4/L5 level, which affected the detailed display of the surrounding anatomical structure. In addition, surgery interferes with the normal anatomical structure, further increasing the difficulty of MRI observation of nerve root movement and dural sac compression at the operative level. The continuous scanning and fat suppression of MRM made up for the deficiency of MRI, thus clearly showing the dural sac and nerve root sleeve, which better reflects the postoperative nerve compression. When measuring the postoperative ISH and ISA, MRI was able to accurately evaluate disc morphology and thus accurately assess the loss of ISH and the curvature of vertebral body in both groups of patients.

During the 2-year follow-up period, patients' recovery was evaluated mainly based on lumbocrural pain and lumbar spine mobility. In both groups, the postoperative pain was significantly relieved, and the lumbar spine mobility was restored. MRM can better display the spinal cord and nerve roots, helping doctors better understand the recovery of patients, so as to develop targeted treatment plans and guide patients to carry out rehabilitation exercise. For those with residual nerve root stimulation, treatment measures such as pain relief, nerve nutrition, and relaxation can be taken to relieve the symptoms of nerve compression. Therefore, MRM helps to better relieve pain and promote the recovery of lumbar spine mobility. Moreover, the 2-year recurrence rate of LDH in the MRI group was significantly higher than that in the MRI + MRM group, with a higher incidence of lumbar instability.

The novelty of this study is that we analyzed and compared the effects of MRI and MRI + MRM in LDH from multidimensional perspectives of nerve root sheath, epidural indentation, ISH, ISA, the degree of low back pain, lumbar functional recovery, and recurrence rate, which confirmed that MRI + MRM was more effective in improving the prognosis of LDH patients undergoing PTED. However, this study has several limitations. First, the sample size is small, and increasing the sample size will help to improve the accuracy of research results. Second, there is a lack of analysis on the prognostic factors affecting LDH patients after PTED. If this analysis can be supplemented, it will help to further improve the prognosis of patients. We will further improve the research from the above perspectives in the future.

## 5. Conclusion

In MRM imaging technology, fast spin echo sequence and fat suppression technology were used, which could fully suppress the signal of fat tissue and other tissues around nerve roots by continuous scanning and sufficiently highlight the long T2 signal of CSF, so as to clearly display the dural sac and nerve root sleeve filled with CSF. This is particularly true for patients after PTED, as surgery can cause disturbance of the normal anatomical structure, which further interferes with MRI observation of nerve roots. On MRM images, the signals such as the morphology and deformation of nerve root sleeve as well as epidural indentation can be well displayed, so as to better evaluate the relief of spinal cord and nerve root compression after operation. Under the guidance of MRM, clinicians can take targeted treatment measures to better relieve postoperative pain, improve lumbar spine mobility, and reduce the recurrence of herniation of the same lumbar process. Therefore, MRM plays an important role in improving the prognosis of LDH patients after PTED.

## Figures and Tables

**Figure 1:** MRI sagittal and axial images (a, b) and MRM images (c, d) of lumbar disc herniation.

**Figure 2:** Observation of nerve root sheath sleeve in terms of morphology and shape sleeve deformation on MRI and MRI + MRM. ^∗^*P* < 0.05.

**Figure 3:** Observation of epidural indentation on MRI and MRI + MRM. (a) Comparison of epidural indentation radius vector between MRI and MRI + MRM. (b) Comparison of epidural indentation longitudinal axis between MRI and MRI + MRM. ^∗^*P* < 0.05.

**Figure 4:** Observation of ISH loss (a) and ISA change (b) on MRI and MRI + MRM within one year after PTED.

**Figure 5:** Pain relief and lumbar function recovery in the MRI and MRI + MRM groups. (a) Comparison of waist pain relief within one year after PTED. (b) Comparison of leg pain relief within one year after PTED. (c) Comparison of lumbar function recovery within one year after PTED. ^∗^*P* < 0.05.

**Figure 6:** The two years' follow-up in the MRI and MRI + MRM groups. (a) Comparison of recurrence of LDH at the operative level. (b) Comparison of lumbar instability at the operative level. ^∗∗^*P* < 0.01.

**Table 1:** Comparison of baseline data between the two groups (*n* (%), $\bar{x}\pm s$).

Baseline date		MRI + MRM group (*n* = 32)	MRI group (*n* = 64)	*t*/*χ*^2^	*P*
Age (years)		49.12 ± 2.23	48.88 ± 3.19	0.378	0.706
Sex (male/female)		21/11	34/30	1.362	0.243
BMI (kg/m^2^)		24.01 ± 2.36	23.68 ± 2.45	0.630	0.530
Course of disease (m)		9.11 ± 1.95	9.28 ± 1.71	-0.438	0.662
Protrusive segment	L4/L5	11 (34.38)	25 (39.06)	0.200	0.655
	L5/S1	21 (65.63)	39 (60.94)		
Prominent types	Central type	16 (50.00)	34 (53.13)	0.448	0.799
	Lateral type	6 (18.75)	14 (21.88)		
	Paracentral type	10 (31.25)	16 (25.00)		

## Data Availability

The simulation experiment data used to support the findings of this study are available from the corresponding author upon request.
